The article "Clinicopathological characteristics and long-term prognosis of screening detected non-palpable breast cancer by ultrasound in hospital-based Chinese population (2001-2014)" was published in 2016. Journal: Oncotarget.

# Clinicopathological characteristics and long-term prognosis of screening detected non-palpable breast cancer by ultrasound in hospital-based Chinese population (2001-2014)

**DOI:** 10.18632/oncotarget.12319

**Published:** 2016-09-28

**Authors:** Bo Pan, Ru Yao, Qing-Li Zhu, Chang-Jun Wang, Shan-Shan You, Jing Zhang, Qian-Qian Xu, Feng Cai, Jie Shi, Yi-Dong Zhou, Feng Mao, Yan Lin, Jing-Hong Guan, Song-Jie Shen, Zhi-Yong Liang, Yu-Xin Jiang, Qiang Sun

**Affiliations:** ^1^ Department of Breast Surgery, Peking Union Medical College Hospital, Chinese Academy of Medical Sciences & Peking Union Medical College, Beijing, P. R. China (100730); ^2^ Department of Ultrasound, Peking Union Medical College Hospital, Chinese Academy of Medical Sciences & Peking Union Medical College, Beijing, P. R. China (100730); ^3^ Department of Radiology, Peking Union Medical College Hospital, Chinese Academy of Medical Sciences & Peking Union Medical College, Beijing, P. R. China (100730); ^4^ Department of Pathology, Peking Union Medical College Hospital, Chinese Academy of Medical Sciences & Peking Union Medical College, Beijing, P. R. China (100730)

**Keywords:** non-palpable breast cancer, screening, ultrasound, prognosis

## Abstract

**Purpose:**

The mainstay modality of breast cancer screening in China is the hospital-based opportunistic screening among asymptomatic self-referred women. There is little data about the ultrasound (US) detected non-palpable breast cancer (NPBC) in Chinese population.

**Methods:**

We analyzed 699 consecutive NPBC from 1.8-2.3 million asymptomatic women from 2001 to 2014, including 572 US-detected NPBC from 3,786 US-positive women and 127 mammography (MG) detected NPBC from 788 MG-positive women. The clinicopathological features, disease-free survival (DFS) and overall survival (OS) were compared between the US- and MG-detected NPBC. Prognostic factors of NPBC were identified.

**Results:**

Compared to MG, US could detect more invasive NPBC (83.6% vs 54.3%, p<0.001), lymph node positive NPBC (19.1% vs 10.2%, p=0.018), lower grade (24.8% vs 16.5%, p<0.001), multifocal (19.2% vs 6.3%, p<0.001), PR positive (71.4% vs 66.9%, p=0.041), Her2 negative (74.3% vs 54.3%, p<0.001), Ki67 high (defined as >14%, 46.3% vs 37.0%, p=0.031) cancers and more NPBC who received chemotherapy (40.7% vs 21.3%, p<0.001). There was no significant difference in 10-year DFS and OS between US-detected vs MG-detected NPBC, DCIS and invasive NPBC. For all NPBC and the US-detected NPBC, the common DFS-predictors included pT, pN, p53 and bilateral cancers.

**Conclusion:**

US could detect more invasive, node-positive, multifocal NPBC in hospital-based asymptomatic Chinese female, who could achieve comparable 10-year DFS and OS as MG-detected NPBC. US would not delay early detection of NPBC with improved cost-effectiveness, thus could serve as the feasible initial imaging modality in hospital-based opportunistic screening among Chinese women.

The article "Clinicopathological characteristics and long-term prognosis of screening detected non-palpable breast cancer by ultrasound in hospital-based Chinese population (2001-2014)" was published in 2016. Journal: Oncotarget.

## INTRODUCTION

Breast cancer is now the most common cancer in Chinese women, and the leading cause of cancer death in women younger than 45 years [1, 2]. Chinese women usually have smaller and denser breasts compared to Caucasian counterparts [1, 3, 4], which would reduce the diagnostic accuracy of mammography (MG) [5]. The younger median age at breast cancer diagnosis in Chinese women compared with females in high-income countries also makes MG less effective in breast cancer detection [6, 7]. Given the huge population in China with its geographic diversity, urban rural disparity, and the demographic epidemiology of developing breast cancer, screening strategy might be different from the annual/biennial mammographic screening in the Western world. The current mainstay modality of breast cancer early detection in China is the hospital-based opportunistic screening among asymptomatic self-referred women.

Milestone studies showed that ultrasound (US) was not only a useful supplementary imaging tool of MG for women with dense breast or elevated risk [8–14], but an effective primary screening test for breast cancer both in the western world and in China [7, 15–18]. US was widely used as initial imaging test for breast detection in hospitals in China, and also designated as the primary screening tool in the standard protocol of the Two Cancers Screening Project jointly launched by the National Health and Family Planning Commission (former Ministry of Health of China) and the All-China Women's Federation [19–22]. However, there is little data about the specific features and prognosis of the US-detected non-palpable breast cancer (NPBC) in hospital-based Chinese population. Thus, we performed this study to compare the clinicopathological characteristics and the long-term survival of US-detected and MG-detected NPBC in Chinese women.

## RESULTS

### Descriptive information of the study cohort

A total of 4,574 patients with positive screening imaging test (defined as BI-RADS 4 and 5) underwent biopsies, including 3,786 US-guided biopsies and 788 MG-guided biopsies as described in METHOD. 729 NPBC were diagnosed with 588 US-detected NPBC and 141 MG-detected NPBC, thus the positive predictive value (PPV) of US-guided biopsy was 15.5% and the PPV of MG-guided biopsy was 17.9%. After excluding 16 US-NPBC patients and 14 MG-NPBC patients whose clinicopathological information were missing, 699 NPBC patients including 572 US-NPBC and 127 MG-NPBC were analyzed in the study, comprising 7.9% of contemporary 8,821 breast cancer treated in PUMC Hospital. 680 patients (97.3%) were treated during the recent ten years (2005-2014) while 551 patients (78.8%) were treated during the recent five years (2010-2014). 462 patients (66.1%) were pre-menopausal and 237 (33.9%) post-menopausal. With a median follow-up time of 36 months (6-163 months, mean 42 months), 32 patients including 27 US-NPBC and 5 MG-NPBC developed recurrence or metastasis. Nine patients who were all detected by US passed away including 6 breast cancer related deaths and 3 deaths due to other cause (Figure 1).

The article "Clinicopathological characteristics and long-term prognosis of screening detected non-palpable breast cancer by ultrasound in hospital-based Chinese population (2001-2014)" was published in 2016. Journal: Oncotarget.

**Figure 1:** Diagram of the research design Asymptomatic Chinese women were screened to detect non-palpable breast cancer (NPBC). The clinic-pathological characteristics, disease free survival (DFS) and overall survival (OS) were compared between ultrasound (US) detected NPBC and mammogram (MG) detected NPBC. DFS and OS related prognostic factors of all NPBC, US-detected and MG-detected NPBC were identified. **A.** The total 1.8-2.4 million asymptomatic women participated in the hospital-based screening was estimated with the 699 screen-detected NPBC and the incidence of 30-40/ten thousand. **B.** The Beijing's Two Cancers Screening Project had screened breast cancer with physical examination (PE) and ultrasound in a combination of community-based and hospital-based manner. Part of the women with positive screening ultrasound cases had been transferred and treated in PUMC Hospital. **C.** Dense breasts were defined as BI-RADS category 3 and 4 (edition 2003), or C and D (edition 2013). **D.** Positive imaging study of US and MG was defined as BI-RADS 4 and 5. **E.** Some women would refuse mammogram due to the minor radioactivity or the extra expensed, or because it would be painful to perform for small breasts. **F.** Negative imaging study of US and MG was defined as BI-RADS 1, 2 and 3.

### Comparison of clinicopathological characteristics between US detected NPBC and MG-detected NPBC

Compared to MG, US could detect more invasive NPBC (83.6% vs 54.3%, p<0.001), lymph node positive cancer (19.1% vs 10.2%, p=0.018), low grade cancer (24.8% vs 16.5%, p<0.001), multifocal cancer (19.2% vs 6.3%, p<0.001), PR positive cancer (71.4% vs 66.9%, p=0.041), Her2 negative cancer (74.3% vs 54.3%, p<0.001), Ki67 high cancer (defined as >14%, 46.3% vs 37.0%, p=0.031) and more NPBC which needed chemotherapy (40.7% vs 21.3%, p<0.001). There was no significant difference between these two groups of NPBC in age, lymphovascular invasion (LVI), laterality, surgery, radiotherapy, and anti-Her2 targeted therapy (Table 1).

The article "Clinicopathological characteristics and long-term prognosis of screening detected non-palpable breast cancer by ultrasound in hospital-based Chinese population (2001-2014)" was published in 2016. Journal: Oncotarget.

**Table 1:** Clinicopathological characteristics of screening-detected NPBC from hospital-based population

Characteristics	No. (%) of Patients		P^a^
	US-NPBC	MG-NPBC	
**Total**	572	127	
**Age (years)**			
**Mean±SD**	51.33±12.67	50.29±11.53	0.396
**Age at diagnosis**			0.065
<40	96 (16.8)	14 (11.0)	
40~49	192 (33.6)	56 (44.1)	
50~59	140 (24.5)	33 (26.0)	
≥60	144 (25.1)	24 (18.9)	
**Tumor histology**			**0.000**
DCIS NPBC	94 (16.4)	58 (45.7)	
Invasive NPBC	478 (83.6)	69 (54.3)	
**pT**			**0.000**
Tis	94 (16.4)	58 (45.7)	
T1a	82 (14.3)	29 (22.8)	
T1b	141 (24.7)	14 (11.0)	
T1c	208 (36.4)	19 (15.0)	
T2	47 (8.2)	7 (5.5)	
**Lymph node status**			**0.018**
Negative	463 (80.9)	114 (89.8)	
Positive	109 (19.1)	13 (10.2)	
**Number of positive LN**			0.378
**Mean±SD**	1.03±3.78	0.70±3.66	
**pN**			0.050
N0	463 (81.0)	114 (89.8)	
N1	74 (12.9)	7 (5.5)	
N2	13 (2.3)	4 (3.1)	
N3	22 (3.8)	2 (1.6)	
**TNM stage^b^**			**0.000**
0	94 (16.4)	58 (45.7)	
Ia	343 (60.0)	53 (41.7)	
Ib	2 (0.3)	0 (0.0)	
IIa	84 (14.7)	7 (5.5)	
IIb	14 (2.6)	3 (2.4)	
IIIa	13 (2.2)	4 (3.1)	
IIIc	22 (3.8)	2 (1.6)	
**Histological grade**			**0.000**
Low grade	142 (24.8)	21 (16.5)	
Medium grade	288 (50.3)	59 (46.5)	
High grade	111 (19.4)	45 (35.4)	
Unknown	31 (5.4)	2 (1.6)	
**Focality**			**0.000**
Monofocal	462 (80.8)	119 (93.7)	
Multifocal	110 (19.2)	8 (6.3)	
**Laterality**			0.187
Unilateral	514 (89.9)	109 (85.8)	
Bilateral	58 (10.1)	18 (14.2)	
**LVI**			0.642
No	546 (95.5)	120 (94.5)	
Yes	26 (4.5)	7 (5.5)	
**ER**			0.052
Negative	129 (22.6)	28 (22.0)	
Positive	441 (77.1)	96 (75.6)	
Unknown	2 (0.3)	3 (2.4)	
**PR**			**0.041**
Negative	162 (28.3)	39 (30.7)	
Positive	408 (71.4)	85 (66.9)	
Unknown	2 (0.3)	3 (2.4)	
**Hormone receptor**			0.051
Negative	114 (19.9)	24 (18.9)	
Positive	456 (79.7)	100 (78.7)	
Unknown	2 (0.3)	3 (2.4)	
**Her2 status**			**0.000**
Negative	425 (74.3)	69 (54.3)	
Positive	92 (16.1)	27 (21.3)	
Unknown	55 (9.6)	31 (24.4)	
**Ki67**			**0.031**
<14%	292 (51.1)	72 (56.7)	
≥14%	265 (46.3)	47 (37.0)	
Unknown	15 (2.6)	8 (6.3)	
**p53**			**0.023**
Negative	392 (68.6)	84 (66.1)	
Positive	169 (29.5)	35 (27.6)	
Unknown	11 (1.9)	8 (6.3)	
**Immunophenotype^c^**			**0.000**
DCIS	94 (16.4)	58 (45.7)	
Luminal A	176 (30.8)	21 (16.6)	
Luminal B	183 (32.1)	30 (23.6)	
Her2	38 (6.6)	5 (3.9)	
TNBC	54 (9.4)	4 (3.1)	
Unknown	27 (4.7)	9 (7.1)	
**Surgery**			0.488
Mastectomy	448 (78.3)	103 (81.1)	
Breast conserving surgery	124 (21.7)	24 (18.9)	
**Chemotherapy**			**0.000**
No	339 (59.3)	100 (78.7)	
Yes	233 (40.7)	27 (21.3)	
**Radiotherapy**			0.476
No	464 (81.1)	100 (78.7)	
Yes	104 (18.2)	27 (21.3)	
Unknown	4 (0.7)	0 (0.0)	
**Anti-Her2 targeted therapy**			0.706
No	503 (88.0)	115 (90.6)	
Yes	58 (10.1)	10 (7.9)	
Unknown	11 (1.9)	2 (1.5)	
**Endocrine therapy**			0.051
No	119 (20.9)	25 (19.7)	
Yes	451 (78.8)	99 (78.0)	
Unknown	2 (0.3)	3 (2.4)	

Abbreviations: NPBC, non-palpable breast cancer; US, ultrasound; MG, mammography; SD, standard deviation; TNM, tumor, node, metastasis system; DCIS, ductal carcinoma *in situ*; ER, estrogen receptor; PR, progesterone receptor; LVI, lymphovascular invasion.

a Bold type indicates statistical significance.

b TNM stage is according to the 7^th^ AJCC cancer staging system.

c Immunophenotype of invasive NPBC is according to the the immunohistochemical subtype of 2013 St. Gallen Consensus.

The article "Clinicopathological characteristics and long-term prognosis of screening detected non-palpable breast cancer by ultrasound in hospital-based Chinese population (2001-2014)" was published in 2016. Journal: Oncotarget.

### Survival outcomes and prognostic factors of NPBC

The 10-year Kaplan-Meier estimated disease free survival (DFS) of all NPBC patients, US-NPBC and MG-NPBC were 91.0%, 90.6% and 92.7%, whereas the 10-year overall survival (OS) were 96.9%, 96.1% and 100.0% respectively. As for the ductal carcinoma *in situ* (DCIS), the 10-year Kaplan-Meier estimated DFS of US-DCIS-NPBC and MG-DCIS-NPBC were 100.0% and 93.8%, whereas the 10-year OS were both 100.0%. The 10-year Kaplan-Meier estimated DFS of invasive US-NPBC and invasive MG- NPBC were 88.6% and 92.0%, whereas the 10-year OS were 95.2% and 100.0% respectively. There was no significant difference in 10-year DFS or OS between US- and MG-detected NPBC, between US- and MG-detected DCIS or between US- and MG-detected invasive NPBC (Figure 2, Table 2).

**Figure 2:** Kaplan-Meier estimated long-term prognosis of NPBC patients There was no significant difference in both DFS and OS between US- and MG-detected NPBC (Figure 2A, 2B), between US- and MG-detected ductal carcinoma *in situ* (DCIS, Figure 2C), or between US- and MG-detected invasive NPBC (Figure 2D, 2E). Please note that the figure for comparison of US- vs MG-detected DCIS NPBC was unavailable because the OS of US- and MG-detected DCIS NPBC were both 100%, with all patients alive. The US-detected NPBC could achieve similar 10-year DFS and OS compared to MG-detected counterparts.

**Table 2:** Comparison of the Kaplan-Meier estimated 10-year DFS and OS between US- and MG-NPBC

Patients (No.)	NPBC Group (No.)	10-year DFS (%)	P value	10-year OS (%)	P value
All (699)	US (572)	90.6	0.738	96.1	0.142
	MG (127)	92.7		100.0	
DCIS (152)	US (94)	100.0	0.060	100.0	1.000
	MG (58)	93.8		100.0	
Invasive (547)	US (478)	88.6	0.680	95.2	0.239
	MG (69)	92.0		100.0	

Abbreviations: NPBC, non-palpable breast cancer; US, ultrasound; MG, mammography; DFS, disease free survival; OS, overall survival; DCIS, ductal carcinoma *in situ*.

DFS prognostic factor for both all NPBC included pT (p=0.018), pN (p=0.040), laterality (also bilateral cancers, p<0.001) and p53 status (p=0.010) (Table 3), and these same four factors were also identified as the DFS related factors for US-detected NPBC (Table 4). LVI, ER, PR, hormone receptor status, immunophenotype, chemotherapy and endocrine therapy might be potential DFS predictors for both all NPBC and US-detected NPBC according to univariate analysis. However, these factors were not significant in the multivariate analysis. None of the clinicopathological and treatment factors listed above could serve as MG-NPBC DFS factors, or as OS predictors due to the limited events.

The article "Clinicopathological characteristics and long-term prognosis of screening detected non-palpable breast cancer by ultrasound in hospital-based Chinese population (2001-2014)" was published in 2016. Journal: Oncotarget.

**Table 3:** Univariate and multivariate Cox analysis of DFS related prognostic factors of all NPBC patients

Variables	Univariate^a^	Multivariate^b^	
	P^c^	HR (95% CI)	P^c^
**Screening method**	0.738	2.125 (0.667, 6.770)	0.202
**Age at diagnosis**	0.129	0.897 (0.594, 1.354)	0.605
**Histological type**	0.079	1.174 (0.056, 24.709)	0.918
**pT**	**0.002**	**7.332 (1.416, 37.954)**	**0.018**
**Lymph node status**	**0.000**	1.105 (0.228, 5.531)	0.901
**pN**	**0.000**	**3.840 (1.064, 13.855)**	**0.040**
**TNM stage^d^**	**0.000**	0.350 (0.060, 2.040)	0.243
**Focality**	0.201	1.124 (0.388, 3.257)	0.830
**Laterality**	**0.000**	**6.927 (3.010, 15.941)**	**0.000**
**LVI**	**0.000**	1.793 (0.602, 5.341)	0.294
**ER status**	**0.007**	0.436 (0.093, 2.039)	0.292
**PR status**	**0.002**	**0.326 (0.105, 1.017)**	0.054
**Hormone receptor status**	**0.004**	0.000 (0.000, 3.285E+064)	0.891
**HER2 status**	0.215	0.817 (0.284, 2.345)	0.707
**Ki-67 expression**	0.166	0.830 (0.371, 1.856)	0.650
**p53**	0.431	**0.284 (0.109, 0.741)**	**0.010**
**Surgery**	0.290	0.448 (0.176, 1.138)	0.091
**Immunophenotype**	**0.004**	0.803 (0.452, 1.429)	0.456
**Chemotherapy**	**0.000**	2.648 (0.821, 8.541)	0.103
**Radiotherapy**	0.358	0.385 (0.098, 1.507)	0.170
**Anti-Her2 targeted therapy**	0.139	1.037 (0.269, 3.993)	0.958
**Endocrine therapy**	**0.006**	0.965 (0.174, 5.354)	0.968

Abbreviations: HR, hazard ratio; ER, estrogen receptor; PR, progesterone receptor.

a Kaplan-Meier univariate analysis of all factors.

b Adjusted by Cox proportional hazard regression model including all factors with the method of enter.

c Bold type indicates statistical significance.

d TNM stage is according to the 7^th^ AJCC cancer staging system.

e Immunophenotype of invasive NPBC is according to the the immunohistochemical subtype of 2013 St. Gallen Consensus.

**Table 4:** Univariate and multivariate Cox analysis of DFS related prognostic factors of US-detected NPBC patients

Variables	Univariate^a^	Multivariat^b^	
	P^c^	HR (95% CI)	P^c^
**Age at diagnosis**	0.175	0.998 (0.642, 1.551)	0.993
**Histological type**	0.052	0.745 (0.394, 1.412)	0.367
**pT**	**0.001**	**27.672 (4.873, 157.124)**	**0.000**
**Lymph node status**	**0.000**	0.556 (0.108, 2.857)	0.482
**pN**	**0.000**	**5.771 (1.608, 20.710)**	**0.007**
**TNM stage^d^**	**0.000**	0.238 (0.041, 1.390)	0.238
**Focality**	0.688	0.576 (0.164, 2.016)	0.388
**Laterality**	**0.000**	**9.652 (3.925, 23.735)**	**0.000**
**LVI**	**0.000**	2.387 (0.739, 7.711)	0.146
**ER status**	**0.017**	0.744 (0.117, 4.717)	0.754
**PR status**	**0.017**	1.088 (0.196, 6.049)	0.923
**Hormone receptor status**	**0.002**	0.000 (0.000, 9.542E+051)	0.826
**HER2 status**	0.477	0.748 (0.218, 2.565)	0.644
**Ki-67 expression**	0.309	1.083 (0.457, 2.569)	0.856
**p53**	0.210	**0.241 (0.084, 0.689)**	**0.008**
**Immunophenotype**	**0.002**	0.699 (0.401, 1.218)	0.206
**Surgery**	0.614	0.406 (0.132, 1.252)	0.117
**Chemotherapy**	**0.000**	1.740 (0.545, 5.555)	0.350
**Radiotherapy**	0.585	0.158 (0.023, 1.113)	0.064
**Anti-Her2 targeted therapy**	0.218	0.914 (0.157, 5.313)	0.920
**Endocrine therapy**	**0.004**	0.440 (0.057, 3.419)	0.432

Abbreviations: HR, hazard ratio; ER, estrogen receptor; PR, progesterone receptor.

a Kaplan-Meier univariate analysis of all factors.

b Adjusted by Cox proportional hazard regression model including all factors with the method of enter.

c Bold type indicates statistical significance.

d TNM stage is according to the 7^th^ AJCC cancer staging system.

e Immunophenotype of invasive NPBC is according to the the immunohistochemical subtype of 2013 St. Gallen Consensus.

The article "Clinicopathological characteristics and long-term prognosis of screening detected non-palpable breast cancer by ultrasound in hospital-based Chinese population (2001-2014)" was published in 2016. Journal: Oncotarget.

## DISCUSSION

Breast cancer incidence has increased rapidly in the past two decades and is now the most common cancer among women in China. Given the immense scale of the Chinese population with diversity, study showed that it might take 40 years to screen each woman in the target age group once [2]. The former Ministry of Health of China and All-China Women's Federation jointly launched a 3-year (2009-2011) national project which provided free breast cancer screening for 1.46 million rural women aged 35–59 years [7, 19–22]. The 3-year second phase (2012–2015) of this project was to provide free breast cancer screening for 6 million rural women aged 35–64 years [7, 23]. Six million women was a huge screening cohort, however, it only comprised 0.90% (6 million/667.03 million) of all female in China. With a cross-sectional assumption and estimated with the current breast cancer incidence of 30-40/ten thousand in rural areas of China, there would be approximately 1,800-2,400 screening detected breast cancer to be diagnosed out of these 6 million women in one year. However, it only comprised 0.67%-0.89% (1,800-2,400/268.6 thousand) of all newly-diagnosed female breast cancer in 2015 [2]. In Beijing, Shanghai and other cities in China, medical insurance of various sorts would usually cover most of the expenses when asymptomatic women intentionally ask for breast physical examination and screening imaging tests in hospital. So in the current diversified breast cancer screening in China, hospital-based opportunistic screening among asymptomatic women is still the mainstay measure.

The article "Clinicopathological characteristics and long-term prognosis of screening detected non-palpable breast cancer by ultrasound in hospital-based Chinese population (2001-2014)" was published in 2016. Journal: Oncotarget.

Ultrasound has the advantages of portability, inexpensiveness, nonradioactive and improved sensitivity in women with dense breasts. It is widely accepted that US is an useful supplementary tool for MG in women with dense breast or elevated risk [8–14], Berg WA et al. showed in the ACRIN 6666 trial that adding a single screening US to MG would yield an additional 1.1 to 7.2 breast cancers per 1000 high-risk women, also with increase of the false positives [8]. Kolb TM et al. showed that screening US could depict small, early-stage, MG-occult cancers similar in size and stage to MG-NPBC and smaller and lower in stage than palpable cancers in dense breasts [13]. Similar benefit of US as an adjunct to screening MG was reported in women with increased risk and dense breasts [11] with 15% additional detection of the MG occult breast cancers [14] as well as lethal breast cancers [24]. A systematic review showed that supplemental US in women with dense breast tissue permitted detection of small, otherwise occult breast cancers. Potential adverse impact was increased biopsy rate.

Moreover, US is currently regarded as effective primary screening test for breast cancer [7, 15–18]. Benson SR et al. evaluated US as a first-line diagnostic tool and revealed that US is significantly better than MG for detecting invasive breast cancer [17]. Berg WA et al. pushed the ACRIN 6666 trial to a higher level showing that cancer detection rate with US is comparable with MG, with more invasive and node-negative cancers and more false positives [15, 16]. A small-sample-size prospective double-blind study showed that primary US is capable of detecting NPBC in asymptomatic women at an early stage with acceptable rate of false positive [18]. In our previous studies, we showed with a multi-center randomized controlled trial that US would be the preferred imaging test for breast cancer screening in high risk Chinese women [7], and be more sensitive than MG (100.0% vs 57.1%, P=0.04) with improved diagnostic accuracy (0.999 vs 0.766, P=0.01). There was no difference between MG and US in specificity (100% vs 99.9%, P=0.51) and PPV (72.7% vs 70.0%; P=0.87). US would cost approximately $20-30USD while MG cost $65-75USD. To detect one breast cancer, the costs of US, MG, and combined modality were $7876, $45,253, and $21,599 USD, respectively [7]. Thus, although MG is still recommend as the initial/primary imaging test for breast cancer screening according to the Chinese Anti-Cancer Association Guidelines [25], US had been officially designated to be the initial imaging test for breast cancer screening in the national ‘Two Cancer Screening’ campaign in China [7, 26]. However, few studies had reported clinical and pathological features of US-detected NPBC as well as its long term survival prognosis.

The article "Clinicopathological characteristics and long-term prognosis of screening detected non-palpable breast cancer by ultrasound in hospital-based Chinese population (2001-2014)" was published in 2016. Journal: Oncotarget.

Screen-detected breast cancers could occasionally be palpable in patients unaware of the symptom, however, most of the screen-detected cancers are NPBC in asymptomatic women. Although there are concerns about over-diagnosis of screen-detected NPBC based on natural history observation cohort study that some breast cancer might regress or never progress [27, 28], the association between screen-detected DCIS and subsequent invasive interval cancers suggests that detection and treatment of DCIS is still worthwhile in prevention of future invasive disease [29]. Currently the treatment strategy of NPBC is made according to palpable cancers of similar stage, subtype and grade [30]. Bae MS et al. reported comparison study between 807 MG-detected NPBC vs 256 US-detected NPBC [31]. However, the 807 (MG+/US not done) NPBC would include some MG+/US- NPBC and majority of MG+/US+ NPBC patients, while the 256 US-detected NPBC patients were all MG-/US+. Similarly in our study, there would also be MG+/US+ double positive NPBC patients in the (US+/MG not done) group. Factors of early detection level such as pT and pN stage were identified as DFS predictors instead of factors revealing disease nature such as the molecular subtype. Laterality was also identified as DFS factors because the contralateral breast cancer might not be NPBC and thus affect the survival. Overall, US could detect more invasive, lymph node positive, low grade tumor, multifocal cancer and still the survival results showed no difference between US and MG detected NPBC. This might explained by the more intensive treatment. For example, there were significantly more US-NPBC patients received chemotherapy (40.7% vs 21.3%, p<0.001).

There are several limitations in our study. Firstly, there is no uniform national breast cancer screening currently in China, and patients with positive US were screened by multi-modalities. So there was no data about the estimated 1.8-2.4 million women out of whom these NPBC patients were diagnosed. Secondly, there were NPBC patients detected by both US and MG who did not have dense breasts, and NPBC patients detected by US only but did not receive MG. These NPBC were all counted as US-NPBC, however, a small portion of these NPBC could also be visualized by MG. Thirdly, it seemed to make more sense to compare NPBC only detected by US versus NPBC only detected by MG. However, NPBC only detected by US but not by MG was difficult to identify and such comparison would exclude patients with dense breasts who did not receive mammogram. Fourthly, in our study cohort, there supposed to be more women with elevated risk such as family history of cancer, previous breast biopsy for benign diseases or hormone replacement therapy, and more women of more advantageous socioeconomic status and easy access to medical resources. This would result in selection bias. Last but not the least, it was a retrospective non-randomized single-center study with limited case number and follow-up time, so there were not enough OS events to identify OS prognostic factors.

The article "Clinicopathological characteristics and long-term prognosis of screening detected non-palpable breast cancer by ultrasound in hospital-based Chinese population (2001-2014)" was published in 2016. Journal: Oncotarget.

In conclusion, our study revealed that compared to MG, US could detect more invasive, node-positive, multifocal NPBC as initial screening test in hospital-based asymptomatic Chinese women, who could achieve comparable 10-year DFS and OS of MG-detected NPBC. US would not delay the early detection of NPBC with improved cost-effectiveness, and thus could serve as the feasible primary imaging modality in hospital-based opportunistic screening among Chinese women.

## MATERIALS AND METHODS

### Ethics statement

This study was approved by the Ethics Committee of the Peking Union Medical College Hospital, Chinese Academy of Medical Sciences.

### Patient selection, pathology review and follow-up

From January 2001 to December 2014, 4,574 asymptomatic patients with positive screening imaging US or MG (defined as BI-RADS 4 and 5) underwent biopsies in PUMC Hospital according to the medical records searching. These “screening positive” patients included self-referred women who came to PUMC Hospital, other hospitals or healthcare institutions in China for opportunistic screening and later came to the breast clinics in PUMC Hospital as “screening positive” for biopsy or surgery. Women enrolled in this study were all self-referred without randomization and asymptomatic without palpable breast mass or nipple discharge. Other “screening positive” patients were women enrolled in the community-based Two Cancer Screening Project in Beijing and in China [20, 21, 23] and transferred to PUMC Hospital with the positive finding. About 1/3 of the patients were local from Beijing, and the other 2/3 from other provinces in China. US-guided biopsy was performed for the US positive patients, regardless of the result of mammogram while MG-guided biopsy was performed only for the MG-positive US-negative patients (Figure 1). 729 NPBC were diagnosed with 588 US-detected NPBC and 141 MG-detected NPBC out of a total 1.8-2.4 million asymptomatic women participated in the hospital-based screening estimated with the breast cancer incidence of 30-40/ten thousand in rural areas of China [2]. All NPBC patients' formalin-fixed paraffin-embedded (FFPE) pathological sections were reviewed to confirm the diagnosis. All patients were followed by telephone call, by out-patient clinics records of follow-up examinations or by both measures. 30 patients including 16 US-NPBC and 14 MG-NPBC were excluded due to missing clinicopathological data. The clinicopathological characteristics, treatment choice, DFS and OS were compared between US-detected NPBC and MG-detected NPBC (Table 1) and the prognostic factors were identified respectively (Table 3, 4, Figure 2).

The article "Clinicopathological characteristics and long-term prognosis of screening detected non-palpable breast cancer by ultrasound in hospital-based Chinese population (2001-2014)" was published in 2016. Journal: Oncotarget.

### Statistical analysis

The quantitative variables were compared with t-test and the categorical variables were compared with chi-square tests. Survival outcomes including 10-year predicted DFS and OS were analyzed and compared by the Kaplan-Meier curve method. Kaplan-Meier univariate analyses and Cox multivariate analyses were performed to identify the DFS and OS prognostic factors for all NPBC, US-detected NPBC and MG-detected NPBC respectively. The significance threshold was set at p<0.05. SPSS software, version 18.0 (SPSS, Inc. Chicago, IL, US) was used for all of the statistical analyses.
